# Clinical Indications for Extubation in Coma Patients with Severe Neurological Craniocerebral Injury with Meta-Analysis

This article has been retracted.

**DOI:** 10.1155/2022/8012018

**Published:** 2022-09-19

**Authors:** Huanhuan Ma, Zhixia Han, Wenlong He, Guowei Liu

**Affiliations:** ^1^Xinxiang Central Hospital, The Fourth Clinical College of Xinxiang Medical University, Xinxiang Henan 453000, China; ^2^School of Public Health, Southwest Medical University, Luzhou Sichuan 646000, China

## Abstract

Computer searches of the PubMed, Cochrane Library, and Embase databases for randomized controlled studies on the effects of intensive nutrition on clinical outcomes in patients with severe craniocerebral injury were conducted from the time of database creation to June 11, 2022, along with manual searches of the relevant literature. Two investigators independently screened the literature, extracted data, and evaluated the risk of bias of the included studies before the effect sizes were combined using RevMan 5.3 statistical software provided by the Cochrane Collaboration Network, and publication bias was detected using Stata 12.0 software. Meta-analysis showed that total protein levels were higher in the intensive nutrition group than in the regular nutrition group (WMD = 4.96 g/L (1.57-8.34), *P* < 0.001); IgA levels were significantly higher in the intensive nutrition group than in the regular nutrition group (SMD = 0.79 (0.51-1.07), *P* < 0.001; SMD = 0.98 (0.58-1.38), *P* < 0.001); IgG levels were significantly higher in the fortified group than in the regular group (SMD = 0.98 (0.58-1.38), *P* < 0.001); CD4/CD8 was significantly higher in the fortified patients than in the regular patients with a combined effect size of WMD = 0.33 (0.18-0.48) (*P* < RR = 0.45 (0.27-0.75), *P* = 0.002). The results show that effective support of early enteral nutrition can reduce the occurrence of gastrointestinal complications in patients, give them a better adaptation process to the gastrointestinal tract, and ensure the degree of tolerance of their gastric mucosa, thus absorbing more nutrition. Fortification significantly reduced the incidence of gastric retention in patients with craniocerebral injury (RR = 0.19 (0.07-0.49), *P* < 0.001). In the subgroup analysis of the three groups, it was shown that, depending on the starting time, the total protein level and IgG level were better in the early nutrition at 24 h than in the late nutrition above 24h and that, depending on the starting dose, the total protein level, IgA, IgG, and CD4/CD8 were better in the intervention at doses above 30 mL/h, using the starting dose of 30 mL/h as the cut-off point. In the subgroup analysis based on different nutrition methods (enteral and parenteral nutrition), IgA levels and the incidence of bloating and diarrhea were better than those of parenteral nutrition in the indicators of enteral nutrition.

## 1. Introduction

Severe traumatic brain injury (STBI) is a common neurosurgical condition that is caused by direct or indirect violence to the head [1], and the Glasgow Coma Scale (GCS) stipulates that a person who is in a coma for more than 6 h or in a coma again after an injury is considered to be in severe traumatic brain injury (STBI). Severe traumatic brain injury (STBI) is a common acute and critical condition in neurosurgery [2, 3]. Severe traumatic brain injury accounts for 13%-21% of craniocerebral injuries and is characterized by critical and dangerous conditions, complexity, high mortality rate, and poor prognosis [4–6]. Patients with severe craniocerebral injury all have different degrees of coma, cannot eat on their own, and have a significant metabolic response to systemic stress, resulting in impaired nutritional intake, metabolic disorders, and depletion of the body's original nutritional reserves, leading to varying degrees of malnutrition soon after admission to the hospital [7]. Enteral nutrition (EN) are usually used in clinical practice, while PN is the intravenous supply of nutrients required by the patient, and EN is the gastrointestinal supply of metabolically necessary nutrients and various other nutrients [8]. The PN is the intravenous supply of nutrients needed by the patient, while the EN is the gastrointestinal supply of metabolically required nutrients and other nutrients [8, 9]. Active and rational nutritional support can improve the overall treatment of the disease and improve the prognosis. With the recognition of PN complications and gastrointestinal stress dysfunction, EN, especially early enteral nutrition, is gaining attention and has even become the first choice for surgical nutritional support [10].

Therefore, while early/late enteral nutrition is strictly limited, the dosage limit should be controlled accordingly. In 2012, the European and American guidelines on surgical nutrition were interpreted [11], and it was suggested that because the gastrointestinal tract of critically ill patients has a gradual process of adaptation and tolerance to enteral nutrition, so when enteral nutrition is implemented in the early stage, it is necessary to start with a small dose and gradually increase the corresponding dose to meet the patient's daily energy requirement. The guidelines recommend that small doses should start from 20 to 50 mL/h and large doses from 100 to 120 mL/h to meet the daily energy requirement. Although enteral nutrition support is currently the most commonly used adjuvant therapy in the clinical treatment of severe craniocerebral injury, the patient's gastrointestinal tract is hypoperfused, which reduces the function of the gastrointestinal tract and prevents the patient from absorbing nutrients properly. Fortified nutrition can effectively improve the gastrointestinal flora, thus providing protection to the gastrointestinal mucosal barrier and improving the immunity of the body [12]. Fortified nutrition means the addition of additional nutrients to the original general nutritional support, called fortified nutrition, which is fortified with nutrients such as glutamine, alanylglutamine, probiotics, and arginine. The purpose of fortification is to enable people to obtain a higher level of comprehensive and reasonable nutritional satisfaction and maintain a higher level of health needs under the normal demands of physiological life and labor. Its important significance and role is to make up for the deficiencies of natural food ingredients, supplement the loss of food nutrients, apply to the needs of special groups and special occupations, and also standardize the reduction of nutritional deficiency diseases or complications caused by nutritional deficiencies, which can effectively save considerable medical costs for the country.

Although the importance of nutritional support is unquestionable, the clinical effect of enteral nutrition can be reduced by different feeding methods of enteral nutrition. The study was selected in terms of language, and only Chinese and English literature was searched, which will have incomplete literature inclusion. The total number of literature included in this study was 39 articles with 3165 study subjects, which still makes it difficult to achieve a large sample for observational analysis. Due to the insufficient sample size of the included studies and the heterogeneity of the literature included in this study in terms of sample and methodology, there is a large variation in the intensity of the intervention programs that can be studied as well as the duration of the intervention, and the range of interventions for the experimental and control groups is also large, which has an impact on the combined results. The reliability of the combined results is affected to some extent. In the subgroup analysis of the three groups, it was shown that, depending on the starting time, the total protein level and IgG level were better in the early nutrition at 24 h than in the late nutrition above 24 h and that, depending on the starting dose, the total protein level, IgA, IgG, and CD4/CD8 were better in the intervention at doses above 30 mL/h, using the starting dose of 30 mL/h as the cut-off point. In the subgroup analysis based on different nutrition methods (enteral and parenteral nutrition), IgA levels and the incidence of bloating and diarrhea were better than those of parenteral nutrition in the indicators of enteral nutrition.

## 2. Related Work

Severe traumatic brain injury (STBI) mainly refers to brainstem injury, extensive brain contusion, and extensive skull fracture due to multiple causes, and patients with STBI are often unable to eat on their own due to varying degrees of impaired consciousness. Patients with severe injuries rapidly enter a hypermetabolic state, followed by a high catabolic state in which the daily nutritional requirements exceed the normal basal caloric and protein consumption, resulting in a negative nitrogen balance [12]. If energy supplementation is not timely, the chance of being in a high metabolic and low nutritional state increases the susceptibility to infection due to poor immune function and slow wound healing, thus affecting the repair and functional compensation of the central nervous system and increasing the morbidity and mortality of patients [13]. For patients with STBI, tracheotomy and enteral nutrition support within 12~24 hours of admission is more beneficial to the recovery of patients [14]. The quality of the literature was evaluated according to the Cochrane Risk of Bias Assessment Tool.

The purpose of this review is to analyze the current controversial issues such as different starting times, starting doses, and different feeding methods of enteral nutrition, so as to provide a reference basis for the development of clinical nutritional support protocols, improve patient outcomes, and shorten patients' hospital stays [15]. The secretion of metabolic hormones such as adrenocorticotropic hormone, catecholamine and glucagon increases in patients with severe craniocerebral injury, accompanied by an increase in energy demand. Parenteral nutrition cannot meet the energy demand of the body after craniocerebral trauma, coupled with the limitation of fluid input in acute cerebral edema and the occurrence of gastrointestinal dysfunction [16]. The intestine is the central organ of high metabolism after trauma, and the barrier function of the intestinal mucosa becomes impaired under the stress state, and the intestinal bacteria can be displaced through the mucosal barrier and infections can occur.

Without timely nutritional support in the early stage of injury, malnutrition will soon result, which will affect the recovery of disease and neuronal repair, and even increase the rate of disability and death. Enteral nutrition in patients with severe craniocerebral injury can be administered through nasogastric tube, nasoduodenal tube, transnasal jejunal tube, and transgastric/jejunostomy feeding. Among them, the simplest and most commonly used enteral nutrition route that is not sensitive to the osmotic pressure of the nutrition solution is transgastric enteral nutrition, but it is not suitable for patients with poor gastrointestinal motility or impaired emptying [17]. For long-term nutritional support (more than 4 weeks), gastro-/jejunostomy feeding is the preferred method, preferably with continuous infusion by infusion pump for 12-24 hours and uniform feeding rate. In addition, enteral nutrition infusion pump is also suitable for patients with heavy cranial injury with artificial airway to reduce gastric retention, avoid gastrointestinal irritation, and reduce the occurrence of adverse reactions such as abdominal distension [18]. The percutaneous endoscopic gastrostomy/jejunostomy can be left in place for a long time, effectively reducing the rate of detachment and avoiding restriction of movement and pressure on the skin and mucosa of patients [19].

## 3. Materials and Methods

### 3.1. Inclusion and Exclusion Criteria

Subjects involved in the literature met the following criteria: clinically definite diagnosis of heavy craniocerebral injury by cranial CT or MRI, Glasgow coma score of 3 to 8, expected treatment time ≥ 7 d, and any gender. Those in pregnancy and patients with cancer and gastrointestinal injuries, combined with severe multiple injuries and cardiopulmonary insufficiency, were excluded, as shown in Figure 1.

The intervention group was given intensive nutrition, i.e., additional nutrients including glutamine, alanine glutamine, probiotics, *ω*-3 fatty acids, arginine, and dietary fiber on top of the normal nutritional support in the control group. The following are the indicators: nutritional indicators: total serum protein; immunological indicators: IgA, IgG, and CD4/CD8; outcome indicators: morbidity and mortality rate; and adverse reaction indicators: total infection rate, bloating and diarrhea, and gastric retention.

Two investigators independently screened the literature according to inclusion and exclusion criteria and used a predesigned data extraction form to extract relevant information, including (i) basic characteristics of the study: first author's name, year of publication, country, and sample size; (ii) basic characteristics of the study population: mean age, male proportion, and mean GCS score; (iii) information related to the intervention: type of fortification, nutrition mode, nutrition initiation time, nutrition initiation dose, feeding route, feeding method, and nutrition duration; and (iv) outcome indicators: total protein level, IgA, IgG, CD4/CD8, morbidity and mortality rate, total infection rate, incidence of bloating and diarrhea, and incidence of gastric retention. The investigators cross-checked the extracted information one by one and resolved any disagreement through discussion or consultation with a third party; if the information material of the study was incomplete, the authors were contacted to obtain relevant information; if no relevant data were obtained, the literature was excluded.

For each of the included studies, each entry was assessed according to the above 7 criteria and evaluated according to “low risk,” “unclear,” and “high risk” criteria. “Low risk” indicates low bias, representing a low risk of bias; “unclear” is moderate bias, indicating a lack of information to determine the level of risk or unclear bias; “high bias “ is a high level of bias, indicating a high risk of a bias. This work was evaluated independently by two investigators, two of whom were the investigator himself and one doctoral student, both of whom were trained in statistics and related professions and both of whom had the ability to complete quality evaluation independently and to discuss or consult a third party to resolve any disputes about the evaluation findings when they existed.

Effect sizes were combined using RevMan 5.3 statistical software provided by the Cochrane Collaboration Network. Categorical variables were analyzed using relative risk (RR), and continuous data were analyzed using mean difference (MD) or standardized mean difference (SMD), and 95% confidence intervals (CI) were calculated for each effect size. The random-effects model was used to combine the effect sizes. In addition, subgroup analyses of study outcome indicators were performed according to the time of initiation (early nutrition (within 24 h) and late nutrition (more than 24 h)), starting dose (small dose (<30 mL/h) and large dose (≥30 mL/h)), and feeding method (pump-in and drip). Stata 12.0 software was used to detect publication bias, and *P* values for both Begg's test and Egger's test > 0.05 suggested no publication bias; *P* ≤ 0.05 suggested publication bias.

### 3.2. Literature Search Results

Based on the search strategy, a total of 960 relevant papers were searched, including 450 in PubMed, 317 in Embase, 49 in Cochrane Library, 75 in Wanfang database, and 69 in CNKI database, and 699 papers were screened for reading abstracts after deleting 261 duplicate papers. The remaining 73 papers were read in full text, and finally, 39 papers were included in this study, as shown in Figure 2.

The basic characteristics of the included study subjects and the interventions are shown in Figure 3. All 39 included papers used a randomized group design, 10 papers used random assignment concealment, 7 papers were blinded to study subjects or investigators, 4 papers were blinded to the outcome analysis process, all 39 papers reported complete results, 33 papers had no selective reporting bias, and 33 papers had no other bias.

### 3.3. Meta-Analysis Results

Random-effects model was used to combine the results, which showed that the total protein levels in the patients with intensive nutrition intervention were higher than those in the regular nutrition group, and the difference was statistically significant (WMD = 4.96 g/L (1.57-8.34), *P* < 0.001), as shown in Figure 4. The cut-off point was 24 h. Nutritional support given within 24 h was defined as early nutrition and beyond 24 h as late nutrition, depending on the onset of nutritional support. Based on the time of initiation, subgroup analyses were performed for the outcome indicators of total protein, IgA, IgG, CD4/CD8, morbidity and mortality, total infection rate, incidence of bloating and diarrhea, and incidence of gastric retention.

Fifteen papers evaluated the effect of fortification interventions on IgA levels. 15 papers evaluated the effect of fortification on IgG levels, and due to the inclusion of different units of IgA in the literature, the combined effect sizes were standardized mean difference (SMD). The heterogeneity test result *I*^2^ = 79%; *P* < 0.001, suggesting a significant heterogeneity. The difference was statistically significant (*P* < 0.001), as shown in Figure 5.

The results of the subgroup analysis showed that early nutrition was better than late nutrition in terms of total protein levels (WMD: 7.34 g/L vs. 3.46 g/L) and IgG levels (SMD: 0.95 vs. 0.89), and the incidence of bloating and diarrhea was lower (RR: 0.42 vs. 0.45) for patients with craniocerebral injury treated with intensive nutrition. Conversely, late nutritional support IgA levels (SMD: 0.89 vs. 0.56) were higher than early nutritional support and had a lower incidence of morbidity and mortality (RR: 0.38 vs. 0.75), total infection rate (RR: 0.40 vs. 0.49), and gastric retention (RR: 0.19 vs. 0.27), as shown in Figure 6. In contrast, small doses of enteral nutrition can reduce the gastrointestinal motility burden and improve gastrointestinal tolerance in critically ill patients due to its small dose; its nourishing effect will maintain the structure and integrity of intestinal mucosa, reduce bacterial translocation and related infections, and thus promote the recovery of gastrointestinal and other organ functions.

However, it was more effective than the starting low-dose intervention in terms of total protein levels. However, the effect of the initial low-dose intervention was better than the initial high-dose intervention in terms of total infection rate (RR: 0.39 vs. 0.59), bloating and diarrhea (RR: 0.40 vs. 0.43), and gastric retention (RR: 0.43 vs. 0.04). The results of the subgroup analysis, based on the different nutrition methods (enteral and parenteral nutrition), suggested that IgA levels were higher with enteral fortification than with parenteral nutrition (SMD: 0.85 vs. 0.57), and the incidence of bloating and diarrhea (RR: 0.43 vs. 0.63) was lower than with parenteral nutrition, while total protein levels (WMD: 9.27 vs. 4.27), IgG (SMD: 1.36 vs. 0.87), and CD4/CD8 (SMD: 1.03 vs. 0.54) were higher than enteral nutrition, and the morbidity and mortality rate (RR: 0.31 vs. 0.51) and total infection rate (RR: 0.31 vs. 0.50) were lower than enteral nutrition.

## 4. Discussion

However, heavy craniocerebral injury can cause serious impairment of consciousness, which leads to difficulties in eating and causes gastrointestinal digestive disorders, resulting in insufficient nutritional intake of the body, which hinders the recovery of the body state. Studies have shown that early enteral nutrition support for patients with severe craniocerebral injury can improve immunity and promote recovery of trauma and neurological function. It has also been shown that fortified nutrition can be a better way to provide adequate nutrition for patients with heavy craniocerebral injury. The use of fortified nutrition combined with early enteral nutrition support for patients with heavy craniocerebral injury can effectively improve the postoperative nutritional status of the body, enhance nutritional support, and have significant effects on the recovery of patients. Depending on the starting dose, the starting small-dose group (starting dose < 30 mL/h) and the starting high-dose group (starting dose ≥ 30 mL/h) were divided. Subgroup analysis showed that the starting high-dose intensive nutritional support was more effective than the starting low-dose intervention in terms of total protein levels (WMD: 2.67 vs. 1.29), IgA (SMD: 0.59 vs. 0.39), IgG (SMD: 0.99 vs. 0.69), and CD4/CD8 (SMD: 0.45 vs. 0.43).

Therefore, in the evaluation of postoperative recovery of patients with severe craniocerebral injury who have implemented intensive nutrition, the assessment of immune indicators is an essential part, which can visually present the postoperative recovery of patients, and we also found that early enteral nutrition implemented with intensive nutrition did recover faster than patients who did not implement intensive nutrition. Therefore, it can be shown that fortification has advantages in improving the nutritional status and promoting the recovery of immune function in patients with severe craniocerebral injury. It also indicates that enteral nutrition with fortification can be an important adjunct to the treatment of patients with severe craniocerebral injury. The results of the analysis showed that the morbidity and mortality rate and infection rate of the intensive nutrition group were significantly lower than those of the general nutrition group, with the morbidity and mortality rate *P* = 0.002 and the infection rate *P* < 0.001, both of which were statistically significant, as shown in Figure 7. Heavy craniocerebral injury is caused by violence or indirect violence leading to extensive skull fracture and brainstem injury in patients, and the treatment of heavy craniocerebral injury is also one of the difficult problems in neurosurgery, with high morbidity and mortality and disability rates. Intensive enteral nutrition can effectively improve the immune function of patients with heavy craniocerebral injury, thus reducing the morbidity and mortality rate and infection rate and promoting the recovery of patients.

The number of patients with gastric retention in the fortified nutrition group was also significantly less than that in the ordinary feeding group, *P* < 0.001, as shown in Figure 8. Patients with severe craniocerebral injury can directly affect patients' feeding and nutrient digestion and absorption due to their heavy injuries, long-term bed rest can trigger malnutrition in patients, perfect and reasonable nutrition measures are crucial in the treatment process, which can better improve patients' prognosis and reduce the occurrence of postoperative complications in patients, and the implementation of intensive nutrition can effectively improve the quality of enteral nutrition care for patients with heavy craniocerebral injury. The temporal subgroup analysis provides an intuitive understanding of the temporal partitioning that allows clinical staff to more effectively use temporal cutoffs when choosing to implement fortification. In recent years, with the accumulation of clinical experience and the continuous development and improvement of neurosurgical emergency medicine, early nutritional support in heavy craniocerebral injury is more and more widely used, and it also shows significant advantages in clinical application; early nutritional support is not only beneficial to the recovery of patients' diseases but also can make heavy craniocerebral injury patients'. Because of the systemic metabolic disorder, increased energy consumption, and accelerated protein decomposition after heavy craniocerebral injury, patients have severe hypoproteinemia, which in turn accelerates the process of brain injury and increases the morbidity and mortality rate; therefore, timely and effective nutritional support is especially important.

In the subgroup analysis of starting low dose and starting high dose, the small-dose group was significantly better than the high-dose group in terms of total infection rate and intervention effect of gastrointestinal complications, while the clinical effect of immune level showed that the clinical effect of the high-dose group was better than that of the small-dose group. Patients with severe craniocerebral injury are often associated with functional impairment of the intestinal mucosa by mechanisms such as ischemia-reperfusion injury, oxidative stress, and inflammatory response mediated by inflammatory transmitters, as shown in Figure 9. Studies have concluded that different doses of intensive nutrition, both small and large doses, can favor the reduction of plasma diamine oxidase while increasing serum glutamine levels to varying degrees, thus effectively promoting intestinal mucosal repair. The 2006 European Nutrition Guidelines, 2008 Australian Nutrition Guidelines, and 2009 US Nutrition Guidelines all recommend full-dose early nutrition, but their evidence levels are all weak at the 2012 AGI guidelines (acute gastrointestinal injury), and the 2013 Canadian guidelines for nutrition in critically ill patients do not give clear recommendations on dose. Although there is still a large controversy regarding the dosage application for the implementation of fortification, the issue of dosage is carried far on the basis of whether to implement fortification early, but it is pointed out through multiple investigations that the advantages of small-dose fortification are greater than large-dose starting fortification. The outcome indicators of IgA, morbidity and mortality, total infection rate, and gastric retention were better in late nutrition combined with fortification than in early nutrition.

## 5. Conclusion

It provides a favorable evidence-based basis for clinical practice in this field. The IgA level in the intensive nutrition group was significantly higher than that in the general nutrition group (SMD = 0.79 (0.51-1.07), *P* < 0.001); the IgG level in the intensive nutrition group was higher than that in the general nutrition group (SMD = 0.98 (0.58-1.38), *P* < 0.001); the CD4/CD8 in the intensive nutrition patients was significantly higher than that in the general nutrition group. The combined effect size of patients was WMD = 0.33 (0.18-0.48) (*P* < 0.001); fortified nutrition significantly reduced the morbidity and mortality rate of patients with craniocerebral injury (RR = 0.45 (0.27-0.75), *P* = 0.002); the infection rate in the fortified nutrition group was significantly lower than that in the general nutrition group (RR = 0.48 (0.39-0.61), *P* < 0.001); fortification reduced the incidence of bloating and diarrhea by 55% compared to the general nutrition group (RR = 0.45 (0.35-0.58), *P* < 0.001); fortification significantly reduced the incidence of gastric retention in patients with craniocerebral injury (RR = 0.19 (0.07-0.49), *P* < 0.001). In the subgroup analysis of the three groups, it was shown that, depending on the starting time, the total protein level and IgG level were better in the early nutrition at 24 h than in the late nutrition at more than 24 h and that, depending on the starting dose, the total protein level, IgA, IgG, and CD4/CD8 were better in the intervention at more than 30 mL/h.

## Figures and Tables

**Figure 1:** Inclusion and exclusion criteria.

**Figure 2:** Flow chart of literature screening.

**Figure 3:** Risk of bias chart.

**Figure 4:** Forest plot of the effect of intensive versus general nutrition on total protein levels in patients with craniocerebral injury.

**Figure 5:** Forest plot of the effect of intensive versus general nutrition on IgA levels in patients with craniocerebral injury.

**Figure 6:** Subgroup analysis of the effect of fortified versus regular nutrition at different starting times on the outcome of patients with craniocerebral injury.

**Figure 7:** Morbidity and mortality rates and infection rates in the intensified nutrition group.

**Figure 8:** Prevalence of bloating and diarrhea in the intensive nutrition group.

**Figure 9:** Analysis of complications in patients with severe craniosynostosis.

## Data Availability

The data used to support the findings of this study are available from the corresponding author upon request.
